The article "Rural Acoustic Landscape Analysis Based on Segmentation and Extraction of Spectral Image Feature Information" was retracted in 2024. Reasons: signs of a paper mill; suspected computer-generated content; unreliable results or conclusions; lack of ethics approval or compliance.

# Rural Acoustic Landscape Analysis Based on Segmentation and Extraction of Spectral Image Feature Information

**DOI:** 10.1155/2022/1742711

**Published:** 2022-10-08

**Authors:** Huijun Xiao, Tangsen Huang, Ensong Jiang

**Affiliations:** ^1^School of Tourism and Cultural Industry, Hunan University of Science and Engineering, Yongzhou, 425199 Hunan, China; ^2^School of Information Engineering, Hunan University of Science and Engineering, Yongzhou, 425199 Hunan, China

## Abstract

Spectrogram is an image that can record voice information, which can be analyzed by analyzing the received image. Spectrograms are used in mechanical fault diagnosis systems to answer questions such as the location, type, and extent of the fault. It is the main tool for analyzing vibration parameters. In actual use, there are three types of spectrograms, namely linear amplitude spectrum, logarithmic amplitude spectrum, and self-power spectrum. The ordinate of the linear amplitude spectrum has a clear physical dimension and is the most commonly used. In this paper, the feature extraction information of rural acoustic landscape is mainly carried out through spectral images, which can effectively improve the segmentation efficiency, ensure the integrity of information, and determine the feasibility of establishing acoustic landscape in rural areas. This article aims to study the analysis of rural acoustic landscape in Guilin, Guangxi, based on the segmentation and extraction of spectral image feature information, through the segmentation and extraction of spectral image feature information, and then analyze the advantages and disadvantages of rural acoustic landscape. In this article, the Gabor wavelet filtering method is proposed to filter and analyze the spectral image. Through the detailed analysis of the insect and bird calls of the forest community near the village of Guilin, Guangxi, finally, the satisfaction and attention of the rural villagers to the acoustic landscape are investigated. The experimental results show that the sound of insects and birds reaches the maximum in spring and the minimum in autumn and winter. Moreover, the attention of rural villagers to acoustic landscape is also very high, with satisfaction of 87.12% and attention of 92.68%.

## 1. Introduction

Nowadays, the domestic landscape design mainly stays on the visual landscape, and people's rich feeling seems to be single. In recent years, designers in Japan, Europe, and the United States have explored various perception methods of outsiders while designing landscapes. This approach is also known as an acoustic landscape. It contains time, space, people, activities, and places. People can not only perceive things visually but also perceive the environment by smell, touch, hearing, and taste. The increasingly interactive modern landscape has opened up more new fields and new methods for landscape design. The acoustic landscape is also called acoustic ecology, which mainly studies the relationship between sound, nature, and society. The original sound landscape design is not pure sound design nor is it pure music playback through the integration of an electronic sound system. Acoustic landscape design is a comprehensive and high-level landscape design, an ecological environmental protection activity that people actively protect and make beautiful sounds.

The article "Rural Acoustic Landscape Analysis Based on Segmentation and Extraction of Spectral Image Feature Information" was retracted in 2024. Reasons: signs of a paper mill; suspected computer-generated content; unreliable results or conclusions; lack of ethics approval or compliance.

In this article, the diversity of rural vegetation is explored, and the number of people in the village, educational background, male-to-female ratio, and age are investigated by a questionnaire. It is explained by the villagers' satisfaction, the time of birdsong, the relative amount of information of actions, the time of insects in different seasons, and the frequency of birds and insects. This article takes Guilin villages in Guangxi as a case. A detailed study of acoustic landscape, combined with actual case analysis, guidance, and summary, can provide a theoretical basis for the application of acoustic landscape in rural design. This is very important for the development of rural design and is a valuable topic. This article studies the application of acoustic landscape in the rural design of Guilin, Guangxi, builds a bridge to promote the communication between rural design and residents' entertainment, breaks the barriers of communication between designers and users, and tries to improve courtyard designers' sense of residence. It should pay attention to the geoacoustic landscape, application in regional gardens, and more respect for user needs. In the face of the accelerating development of society, various pollutions ensue, and sound pollution has increasingly affected people's lives, and people are more yearning for a quiet life in the countryside. Therefore, how to recognize sound and make it the highlight of rich landscape design is the focus of this research.

The calculation speed of the algorithm is a key factor for real-time monitoring of infrasound signals. The existing methods mainly focus on how to improve the classification accuracy rate, and the running speed is slow, and cannot be used for real-time monitoring. Li M uses spectral entropy for the feature extraction of infrasound signals. This method combined with the support vector machine algorithm, while effectively extracting signal features, greatly improves the computational efficiency. Li et al. use the feature extraction of the sound spectrum of the infrasound signal, which is slightly deviated from the subject [1]. Phase indexing refers to the problem of restoring the original image only from Fourier transform or other linear transform size. Regarding the phase index problem, Kawamura et al. proposed a robust phase recovery algorithm for various noises and mixed noises. In this way, the phase indexing process is divided into two steps: contour search and detailed search. The robust phase recovery algorithm can perform index enhancement during phase indexing, increase the index range, and increase the probability of successful indexing [2]. The method he proposed can retrieve noise, but cannot analyze the soundscape. The sound source in the natural environment is usually regarded as an externalized auditory object located outside the head. Baumgartner et al. proposed a model designed to predict sound externalization related to the saliency of spectral cues in the free field [3]. This model can be used for the analysis of natural soundscapes. Spectral composers have put forward detailed theoretical suggestions on musical time, but how these ideas affect their music practice is still a very challenging question. Through the analysis of the articles of Gérard Grisey and Kaija Saariaho, Besada and Cánovas showed how the theoretical framework of basic cognitive operations of mixing and anchoring as a basis for complex meaning construction can clarify the complex musical use of timelines by spectral composers [4]. It shows the use of language notation in music, but not in landscape. Recently, deep recurrent neural networks have achieved great success in various machine learning tasks, and have also been applied to sound event detection. Kim and Kim proposed a method based on gated recurrent neural network combined with auditory spectrum characteristics to improve the accuracy of polyphonic sound event detection in multichannel audio [5]. It is mainly based on the research of deep loop neural network on sound and the lack of research on the sound spectrum. In the microphone array technology, the cross-spectrum matrix is used to locate the sound source. Ocker and Pannert re-examined Daniell's method to average the cross-spectrum matrix of sensor signals in the frequency domain. The results show that the average results of this method and Welch method in the time domain are similar, involving the reduction of variance, the correlation between different sources and the location of multiple sources [6]. Ocker and Pannert mainly study the cross-spectrum, which is a bit far from the spectrogram. Zhang et al. studied the detection of traffic incidents from audio signals. Collect real data in long tunnels and mark audio samples based on traffic incidents, including tire rubbing, vehicle crashing, and other background sounds. An effective spectrum feature is proposed for the rapid classification of audio events [7]. Zhang et al.'s main research is to judge the spectral characteristics by sound, and has no application in the soundscape. Ren et al. conducted a questionnaire survey of potential tourists in both Chinese and English to test their expectations for the soundscape. The results show that although the two groups most like natural sounds, compared with English, the Chinese prefer the sounds of nature, livestock, and melody, while the sounds of traffic and industry are less. In terms of sound source preference, the sound categories related to the interaction between human activities and nature are more dominant in English than that in Chinese. In the expectation of the overall soundscape, the function is the most important aspect of the Chinese, and English is the sound feature; like the Chinese, the expected psychological perception of English is related to emotional reactions, rather than basic ecological consciousness [8]. He mainly expressed that people prefer natural sounds, but he did not make more substantive methods and measures. If the beauty of the rural soundscape is studied and analyzed, it will increase people's love for the rural scene.

The article "Rural Acoustic Landscape Analysis Based on Segmentation and Extraction of Spectral Image Feature Information" was retracted in 2024. Reasons: signs of a paper mill; suspected computer-generated content; unreliable results or conclusions; lack of ethics approval or compliance.

The innovation of this article is to carry out research on sound landscape design. First of all, this topic compares and narrates the research summary of sound landscape in foreign countries and ours, and the research found that the development of our country is still in its infancy, and foreign countries already have relatively complete voices. Second, starting from the sound landscape in various fields, analyze contemporary excellent sound landscape experience cases, including literature, ecology, musicology, and other fields. Discover the diversified manifestations of sound landscapes from different types of sound landscapes. Next, focus on studying the temporal and spatial changes of forest sound and color, select typical sound types according to the regular characteristics of temporal and spatial changes, and conduct experiments on subjective evaluation of soundscapes and physiological changes.

## 2. The Method of Constructing Rural Acoustic Landscape

### 2.1. Theoretical Basis for the Application of Acoustic Landscape in the Countryside

Soundscape [9] is different from previous noise control, and is studying the interrelationship between people, hearing, acoustic environment, and society. Acoustic landscape requires natural sound, environment, and ecology. The requirements are relatively high, but in rural areas, this kind of environment is more appropriate and does not require too much decoration, pure natural soundscape. The acoustic landscape pays more attention to the perception of the outside world. Soundscape relies on hearing to perceive the outside world and requires a unique understanding of sound. Acoustic landscapes can help people soothe their minds and stay happy. Embrace and enjoy nature. This is also an important basis for establishing acoustic landscapes in rural areas.

The article "Rural Acoustic Landscape Analysis Based on Segmentation and Extraction of Spectral Image Feature Information" was retracted in 2024. Reasons: signs of a paper mill; suspected computer-generated content; unreliable results or conclusions; lack of ethics approval or compliance.

Space is a three-dimensional virtual body [10]. Once the space is connected with human-specific activities, it becomes a “place,” and the countryside is an activity place closely related to people's daily life. To apply acoustic landscape in rural design reasonably, in addition to fully understanding the concept of acoustic landscape and basic theories of space, place, and countryside, it is also necessary to understand the meaning of rural landscape beauty, the appreciation and cognition of rural landscape beauty, and people's environment in the environment. Psychological activities and perceptual feelings, so as to better appreciate and judge the beauty of the sound landscape in the rural landscape. The soundscape involves many fields, as shown in Figure 1.

### 2.2. Soundscape

(1) The origin of the soundscape concept.

The term “Soundscape” [11] was first proposed by the Finnish geographer Granoe in 1929. This term is similar to “Landscape” and is composed of two roots: “sound” and “scape.” It was not until the end of the 1960s that Canadian composer and music educator R. Malay Shafer first proposed the concept of “acoustic landscape,” which contained the meaning of “landscape captured with ears” or “auditory landscape.”

There are many research levels in the soundscape. Combined with landscape design, most of the research focuses on public living spaces. In the study of the acoustic landscape of the universe, the acoustic landscape of outdoor space, the acoustic landscape research of public space, residential area [12], the acoustic landscape design of waterfront landscape, and the acoustic landscape research of ecological green space park. However, generally speaking, acoustic landscape research in landscape design focuses on outdoor spaces. Moreover, the study of acoustic landscape and urban planning are combined to conduct urban acoustic landscape research, urban space acoustic landscape design, Komachi acoustic landscape design, historical area acoustic landscape research, and scenic area acoustic landscape enhancement research.

(2) Classification of acoustic landscape.

There are many ways to classify the soundscape, which can be divided according to the physical characteristics of the sound, the perceptual characteristics of the sound, the function of the sound, or the emotional color of the sound. The more commonly used is to classify the sound landscape according to the sound object and characteristics of the sound, that is, classification by sound source and classification by function.

The article "Rural Acoustic Landscape Analysis Based on Segmentation and Extraction of Spectral Image Feature Information" was retracted in 2024. Reasons: signs of a paper mill; suspected computer-generated content; unreliable results or conclusions; lack of ethics approval or compliance.

According to the sound source, the sound landscape can be divided into three types: natural sound, artificial sound, and active sound. According to the function, it can be divided into auditory perception effect, response, and effect.

(3) The development history of the application of acoustic landscape in rural landscape.

The “sound” of nature has played a role in the rural landscape since the emergence of the rural landscape. In other words, the application of the “sound” of nature in the rural landscape develops with the development of the rural landscape. However, with the development of the times and the progress of science and technology, the form and application mode of “sound” slowly began to change, from the birdsong in the mountains to the whistle of the car passing by and from the cuckoo in the early morning to the hustle and bustle of the bustling city. With the development of human history, the early application of “sound” in rural landscape began to appear—musical instrument sound [13] and animal sound were slowly introduced into the rural landscape. At the end of the 18th century and the beginning of the 19th century, with the further development of Western science and technology, electric-powered equipment began to appear, which greatly promoted the application of “sound” in rural landscape. With the development of modern microelectronic technology, intelligent equipment with more and more powerful functions and uses has gradually emerged. Although the application of intelligent equipment is still in the primary stage in the current rural landscape, due to the gradual depletion of some rural landscape resources, intelligent equipment has the advantage of saving resources and replacing natural resources. It has great development potential in the application of rural landscape.

### 2.3. Spectrogram

Spectrogram [14] is a speech spectrogram invented in the Second World War. Generally speaking, as long as the time domain signal is long enough, the spectrogram can be obtained by processing the received time domain signal. The actual value of the spectrogram is very strong, and it can reflect the complete information and spectral characteristics of the sound signal. Spectrogram can convert speech signals into digital images, and digital image technology [15] can also be applied to speech processing, so it is called “visual language.”

(1) Introduction to the spectrogram.

The article "Rural Acoustic Landscape Analysis Based on Segmentation and Extraction of Spectral Image Feature Information" was retracted in 2024. Reasons: signs of a paper mill; suspected computer-generated content; unreliable results or conclusions; lack of ethics approval or compliance.

The spectrogram [16] was successfully developed by Bell Laboratories in 1947. Its appearance broke through the limitations of independent analysis in the voice and time domains. The advent of the spectrogram has aroused the interest of Cooper and others in the United States. They successfully developed a “speech playback machine” in the Haskins laboratory, which realized the technology of converting the spectrogram image into speech. This is the production of speech synthesis.

At present, there are many research methods of the spectrogram, mainly including the artificial neural network method [17], support vector machine method, dynamic time adjustment method, and hidden Markov model [18].

(2) The generation principle of the spectrogram.

The realization process of the spectrogram is shown in Figure 2.

Taking human speech as an example, in the realization of the spectrogram, the speech signal must be read for sampling processing, and the obtained sampled signal must be framed and windowed [19], and the window length *L*_win_ is calculated. The formula is as follows:

(1) $$\begin{array}{c} L=\Delta T/\Delta t, \end{array}$$

(2) $$\begin{array}{c} L_{\text{win}}=\text{length}/L. \end{array}$$

Among them, *ΔT* is the total time length of the speech signal, *Δt* is the steady time length of the speech signal, length is the length of the sampling sequence, and the calculation result of the window length is usually within the range of 2^5^–2^10^.

The next step is to perform short-time Fourier transform (STFT), logarithmic calculation and moving window operations on the sampled signal, and then obtain the energy spectral density *W*, and then pseudocolor it, and finally, generate a spectrogram [20]. Suppose *h*(*n*) is the sampling signal in the discrete time domain, *n* is the sampling number, and *m* is the sampling time. The calculation process of the generated spectrogram is as follows: *h*(*n*) STFT formula:

(3) $$\begin{array}{c} H_{n}\left(\omega \right)=\overset{\infty }{\underset{m=-\infty }{\sum }}h\left(m\right)w\left(n-m\right)e^{-j\omega m}, \end{array}$$

where *w*(*n*) is the window function. The discrete time-domain Fourier transform (DTFT) formula of *h*(*n*) is:

(4) $$\begin{array}{c} H\left(n,\omega \right)=\overset{N-1}{\underset{m=0}{\sum }}h_{n}\left(m\right)e^{-j\omega m}. \end{array}$$

Discrete Fourier Transform (DFT) formula:

(5) $$\begin{array}{c} H\left(n,k\right)=\overset{N-1}{\underset{m=0}{\sum }}h_{n}\left(m\right)e^{-j\left(2\pi km\right)/N}\;0\leq k\leq N-1. \end{array}$$

The result of |*H*(*n*, *k*)| is the short-term amplitude spectrum estimation of *h*(*n*). The energy spectral density *V*(*n*, *k*) at time *m* is:

(6) $$\begin{array}{c} V\left(n,k\right)={\left|H\left(n,k\right)\right|}^{2}=H\left(n,k\right)\cdot H^{*}\left(n,k\right), \end{array}$$

where *H*^∗^(*n*, *k*) represents the conjugate of *H*(*n,k*), the decibel form of the energy spectral density function *V*(*n,k*):

(7) $$\begin{array}{c} V\left(n,k\right)\left(\text{d}B\right)=10{\text{Log}}_{10}\left(V\left(n,k\right)\right). \end{array}$$

Use the coordinate system with time as the abscissa and frequency as the ordinate to represent the value of *V*(*n*,*k*), and the gray level is represented by the brightness of brightness. Such an image is the spectrogram of *h*(*n*).

(3) Texture feature extraction based on Gabor wavelet.

The article "Rural Acoustic Landscape Analysis Based on Segmentation and Extraction of Spectral Image Feature Information" was retracted in 2024. Reasons: signs of a paper mill; suspected computer-generated content; unreliable results or conclusions; lack of ethics approval or compliance.

Gabor [21] is an STFT method based on the Gaussian function [22]. To more appropriately illustrate the regionality and scale of texture features, the researchers constructed a texture feature analysis filter based on the Gabor wavelet. It reflects the regionality and proportion of the texture. The next formula is the high-spherical wavelet formula of the trigonometric function with Gaussian function added:

(8) $$\begin{array}{c} S\left(t,t_{0},s\right)={\text{e}}^{-\sigma {\left(t-t_{0}\right)}^{2}}{\text{e}}^{js\left(t-t_{0}\right)}. \end{array}$$

From equation (8), the Gabor wavelet transform can be defined:

(9) $$\begin{array}{c} H\left(x\left(t\right),t_{0},s\right)=\int_{-\infty }^{\infty }x\left(t\right)S\left(t,t_{0},s\right)\text{d}t. \end{array}$$

Substituting formula (8) into (9), we can get:

(10) $$\begin{array}{c} H\left(x\left(t\right),t_{0},s\right)=\int_{-\infty }^{\infty }x\left(t\right){\text{e}}^{-\sigma {\left(t-t_{0}\right)}^{2}}{\text{e}}^{js\left(t-t_{0}\right)}\text{d}t. \end{array}$$

Expand equation (10) to get:

(11) $$\begin{array}{c} H\left(x\left(t\right),t_{0},s\right)=\int_{-\infty }^{\infty }x\left(t\right){\text{e}}^{-\sigma {\left(t-t_{0}\right)}^{2}}\cos\left(s\left(t-t_{0}\right)\right)\text{d}t+i\int_{-\infty }^{\infty }x\left(t\right){\text{e}}^{-\sigma {\left(t-t_{0}\right)}^{2}}\sin\left(s\left(t-t_{0}\right)\right)\text{d}t. \end{array}$$

The complex number *H*(*x*(*t*), *t*_0_, *s*) obtained by the above formula represents the frequency information of the signal *x*(*t*) at the frequency of *w* and the time of *t*_0_. Of course, this complex number can also be expressed in the form of real and imaginary parts:

(12) $$\begin{array}{c} H\left(x\left(t\right),t_{0},s\right)=a_{\text{real}}+{ia}_{\text{imag}}. \end{array}$$

In addition, polar coordinates can also be used to represent the hypothetical amplitude *a* and the phase angle *ϕ*.

(13) $$\begin{array}{c} a=\sqrt{{a_{\text{real}}}^{2}+{a_{\text{imag}}}^{2}}, \end{array}$$

(14) $$\begin{array}{c} \varphi =\arctan\left(a_{\text{imag}}/a_{\text{real}}\right). \end{array}$$

The article "Rural Acoustic Landscape Analysis Based on Segmentation and Extraction of Spectral Image Feature Information" was retracted in 2024. Reasons: signs of a paper mill; suspected computer-generated content; unreliable results or conclusions; lack of ethics approval or compliance.

### 2.4. Fundamentals of Graph Theory

(1) Basic concepts of graph theory.

The graph in graph theory [23] is an abstract tool for people to portray the connections between concrete things.

The composition of a graph includes a set *V* of objects called vertices or nodes, and a set *E* of objects called edges or elements, denoted as *G* = (*V*, *E*). If *V* and *E* are empty, then *G* is an empty graph, denoted by *φ*. If and only if the sets *E* and *V* are finite, that is, *E* and *V* contain finite edges and vertices, the graph *G* = (*V*, *E*) is said to be finite.

Set *E* can be regarded as a binary relationship on set *V*. Let *V* = {*v*_1_, *v*_2_, ⋯, *v*_*n*_}, the edge (*v*_1_, *v*_2_) is a data member of *E* if and only if there is a connection between *v*_1_ and *v*_1_ under a certain clear definition. If “*v*_1_ to *v*_2_ connection” is equivalent to “*v*_2_ to *v*_1_ connection,” side (*v*_1_, *v*_2_) is the same as side (*v*_1_, *v*_2_), then this side is said to be undirected. If all edges in the graph are undirected, the graph is an undirected graph; otherwise, it is a directed graph. The finite undirected graph is used in the article, and Figure 3(a) is a simple undirected graph.

In the figure, there are no intersections between edges except for vertices, and each side has and only two vertices. Another way to express a graph is the adjacency matrix. Use *n*-order square matrix *A* = (*a*_*ij*_) to store the weight of the edge in graph *G* starting from *v*_1_ and ending with *v*_2_. When there is no connection between two points, it is recorded as 0, and this matrix is called the adjacency matrix of *G*. The adjacency matrix representation of the graph in Figure 3(a) is shown in Figure 3(b).

Generally, suppose vertex *V* = {*v*_1_, *v*_2_, ..., *v*_*n*_} define the similarity of two sample points *v_j_* and *v_i_* as *p_ij_*, use Gaussian similarity function to define the weight between the two vertices, the calculation is shown in formula (15):

(15) $$\begin{array}{c} p_{ij}=\exp\left(-{\left\|v_{i}-v_{j}\right\|}^{2}/2\sigma^{2}\right). \end{array}$$

Among them, *σ* is the scale parameter. In spectral clustering, the commonly used connection graphs mainly include an *ε*-adjacent connection graph and a fully connected graph. The *ε* neighbor connection graph means that when the distance between two vertices is less than *ε*, it is considered that there is a connection between the two vertices, and the weight *p_ij_* is calculated according to formula (15); otherwise, there is no connection, and *p_ij_* is 0. A fully connected graph considers that there are connections between all vertices *v_i_* and *v_j_*.

(2) Matrix representation of the graph.

The article "Rural Acoustic Landscape Analysis Based on Segmentation and Extraction of Spectral Image Feature Information" was retracted in 2024. Reasons: signs of a paper mill; suspected computer-generated content; unreliable results or conclusions; lack of ethics approval or compliance.

Let *G* = (*V*, *E*) be an undirected fully connected graph, the set of vertices is *V* = {*v*_1_, *v*_2_, ..., *v*_*n*_}, the connection weight between vertices *v*_*i*_ and *v*_*j*_ is *p*_*ij*_, which constitutes the weight adjacency matrix *P*(1, 2),*P* = (*p*_*ij*_)(*i*, *j* = 1, 2, ..., *n*), and *p*_*ij*_ = *p*_*ji*_. Define the degree of vertex *v* ∈ *V* as the sum of the connection weights of all associated vertices:

(16) $$\begin{array}{c} d_{i}=\underset{i}{\sum }p_{ij},j\in adjacent\left(i\right). \end{array}$$

The diagonal matrix formed by *d*_1_, *d*_2_, ..., *d*_*n*_ is the degree matrix *W*:

(17) $$\begin{array}{c} W=\left[\begin{array}{cccc} d_{1} & 0 & \cdots & 0\\ 0 & d_{2} & \cdots & 0\\ \vdots & \vdots & \ddots & \vdots \\ 0 & 0 & \cdots & d_{n} \end{array}\right]. \end{array}$$

Given a subset A containing some vertices, *A* ⊂ *V*, its complement is denoted as *A*. Define the $\bar{A}$ indicator vector *l*_*A*_, *l*_*A*_ = (*f*_1_, *f*_2_, ..., *f*_*n*_) ∈ *R*_*n*_, if *v*_*i*_ ∈ *A*, *f*_*i*_ = 0; otherwise, *f*_*i*_ = 0. |*A*| represents the number of vertices in *A*, and vol(*A*) is equal to the sum of the degrees of all vertices in *A*. These two values are commonly used to measure the size of the subset.

For two sets *A* and *B*, define the similarity function assoc (*A*, *B*) of *A* and *B* to measure the similarity between *A* and *B*:

(18) $$\begin{array}{c} \text{assoc}\left(A,B\right)=\underset{i\in A,j\in B}{\sum }p_{ij}. \end{array}$$

When all vertices in set *A* are only internally connected, assoc (*A*, *A*) = vol(*A*).

(3) Laplacian matrix of graph.

The realization of the spectral clustering algorithm [23] mainly relies on the Laplacian matrix of the graph. In this section, we introduce some Laplacian matrices on undirected weight graph G and their important properties. Here, we use the weight adjacency matrix *P* and the degree matrix *W* mentioned in the previous section.

(1) Unnormalized Laplacian matrix L.

The unnormalized Laplacian [24] matrix *L* is defined as equation (19), which is the difference between the degree matrix and the weight adjacency matrix:

(19) $$\begin{array}{c} L=W-P. \end{array}$$

Due to the symmetry of the weight adjacency matrix *W*, *L* is also a symmetric matrix [25]. It is found through research that under normal circumstances *L* is a positive semidefinite matrix, which means that *L* has n non-negative real eigenvalues, and the smallest eigenvalue should be 0, corresponding to an eigenvector of all ones. For the vector *f* ∈ *R*^*n*^, satisfy:

(20) $$\begin{array}{c} f^{\prime }Lf=\frac{1}{2}\overset{n}{\underset{i,j=1}{\sum }}p_{ij}{\left(f_{i}-f_{j}\right)}^{2}. \end{array}$$

(2) Normalized Laplacian matrix *L*_sym_ and *L*_rm_.

The article "Rural Acoustic Landscape Analysis Based on Segmentation and Extraction of Spectral Image Feature Information" was retracted in 2024. Reasons: signs of a paper mill; suspected computer-generated content; unreliable results or conclusions; lack of ethics approval or compliance.

There are two forms of the normalized Laplacian matrix, which are defined as follows:

(21) $$\begin{array}{c} L_{\mathrm{sym}}=W^{-1/2}{LW}^{-1/2}=I-W^{-1/2}{PW}^{-1/2}, \end{array}$$

(22) $$\begin{array}{c} L_{\text{rm}}=W^{-1}L=I-W^{-1}P. \end{array}$$

And, satisfy *L*_sym_ = *W*^1/2^*L*_rm_*W*^−1/2^ between the two.

*L*_sym_ and *L*_rm_ are the same as *L*, both are positive semidefinite matrices [26]. When *λ* is the eigenvalue of *L*_rm_, it is also the eigenvalue of *L*_sym_, *λ* corresponds to the eigenvector of *L*_sym_ as *v*, and the eigenvector corresponding to *L*_rm_ is *p* = *W*^1/2^*v*, and *λ* and *v* satisfy *Lv* = *λWv*. Both *L*_sym_ and *L*_rm_ are used to express by *L*_*n*_, for the vector *f* ∈ *R*^*n*^, it satisfies:

(23) $$\begin{array}{c} f^{\prime }L_{n}f=\frac{1}{2}\overset{n}{\underset{i,j=1}{\sum }}p_{ij}{\left(\frac{f_{i}}{\sqrt{d_{i}}}-\frac{f_{j}}{\sqrt{d_{j}}}\right)}^{2}. \end{array}$$

The three Laplacian matrices introduced above are all used in actual calculations, and the calculations should be analyzed and selected according to the actual situation.

## 3. Experiment on Rural Acoustic Landscape Based on Language Spectrum

The selected address for this experiment is Guilin Village, Guangxi.

### 3.1. Overview of Rural Landscape in Guilin, Guangxi

Famous scenic spots in Guilin, Guangxi, are shown in Figure 4.

These excellent scenic spots have a unique combination of 16 scenic spots and hundreds of scenic spots, as shown in Figure 5.

### 3.2. The Design Conception of the Rural Acoustic Landscape in Guilin

The element of the soundscape [27] is to learn how to choose sound reasonably. In addition to the key point of “listening,” the soundscape also has the visual element of “seeing.” Grasping the overall atmosphere, summarizing and dividing the existing sounds, it is also possible to conceive the sounds that existed many years ago and then disappear now. After investigation, it is found that the local natural sound landscape is rich and man-made noise is less, but only the traditional sound of the countryside, the sound landscape elements are inevitably monotonous, so the following design ideas are drawn. The natural soundscape is mainly designed to enhance people's awareness of environmental protection, establish a historical and cultural area, awaken people's memory of traditional culture, establish a play area, and strengthen the local natural landscape for people to play and learn.

(1) In the natural sound landscape area:

It is recommended to pass through the water landscape as a breakthrough. The sound of water is very rich, the gurgling sound of running water, and the ding-dong sound of spring water. The courtyard can design two water landscape sketches to form regular or irregular sounds. It can also rebuild the natural waterscape of the village, add artificial streams, design a fluid falling water landscape, and design the width of the water area of the falling or flowing water. The time is wide and the time is narrow, or add water-retaining and water-separating stones to control the flow rate and flow of the water to cause different degrees of water sound. Use unused materials to enrich the sound where the water falls, and also make it more visually diverse or highlight the use of the fishing culture concept in the village to design to highlight the difference here, so that people can participate, which can not only enrich the level of the sound landscape but also add a bit of vitality to the quiet village, and it can also help the future. Dispersing the noise can also remind people to increase their awareness of environmental protection.

(2) In the historical and cultural area:

The main reason why the urban and rural landscapes are different is that the rural is more original and localized. It is recommended to use the historical and cultural relics with local characteristics, and the chimneys, cave dwellings with the characteristics of the times, and the processing and transformation of agricultural tools with local cultural characteristics into historical and cultural sound areas, which can strengthen the childhood memories of people who come to play. It can also provide knowledge and broaden their horizons for children who see these cultural relics or sites for the first time. Modern means, such as designing apps, scanning QR codes and other technological means, can be used to artificially reproduce these historical sounds and enrich the sound landscape. It can also become a unique sound landscape of the place, and it can also awaken people's traditional culture.

(3) In the recreation area:

Due to the consideration of funding, you can record some fresh and smart natural sounds, the sound of seawater, the rustle of leaves, the chirping of insects, and the ding-dong sound of running water through speakers or audio equipment, etc. In the leisure square or the seat on the country road, you can also set up artificial birdhouses on the trees where birds like to build nests and install speakers on the birdhouses to amplify the sounds of the birds and allow you to sit down and rest. People feel the peace of mind, which is more in line with the characteristics of rural eco-tourism and strengthens the local natural sound landscape.

(4) In the entertainment area:

Compared with the quietness of other places, the entertainment area should be a slightly lively place. Some landscape sculpture installations can be made. Since it is an entertainment area, it is designed by means of entertainment and interaction. The design is eye-catching, the application of soundscape sketches, the use of imitated soundscapes, the use of local bamboo materials, or the reuse of construction waste materials, and the combination of beautiful sounds and unique shapes can improve the soundscape design. Participation can also be added, and a musical sculpture can be made using the principles of mechanics or acoustics for people to play and learn.

The article "Rural Acoustic Landscape Analysis Based on Segmentation and Extraction of Spectral Image Feature Information" was retracted in 2024. Reasons: signs of a paper mill; suspected computer-generated content; unreliable results or conclusions; lack of ethics approval or compliance.

### 3.3. Questionnaire Survey on the Sound Environment of Guilin Rural Areas

With the current rapid economic development and highly saturated cities, more and more people in cities begin to yearn for the tranquility and beauty of the countryside, and contemporary rural landscape design should become more humane and more focused on experience. To build a more natural rural soundscape, we must first investigate the rural sound environment and explore what needs to be improved.

(1) Questionnaire content.

This questionnaire is designed strictly in accordance with the design principles of the social questionnaire [28], using the scoring method as the main evaluation method, and is divided into 5 evaluation levels.

The questionnaire design of this survey takes “satisfaction” and “importance” as the main evaluation indicators. “Satisfaction” focuses on understanding the respondents' subjective feelings about the sound environment in Guilin's rural areas, and is an important reflection of the quality of the sound environment in Guilin's rural areas; “importance” focuses on how much the interviewee values the sound environment in the residential area. It directly reflects the protection and planning significance of the rural sound environment.

After many field visits, this questionnaire survey sorted out the seven main sound types in the Guilin countryside, including the sound of water, the sound of birds, the sound of insects, the sound of rain, the sound of wind blowing leaves, the sound of car traffic, and the sound of buildings. At the same time, questions such as “please tick the three voices you hear most easily in the surrounding countryside of Guilin,” “rate the voices you want to keep or remove,” and other questions were asked. Based on the interviewee's evaluation of these voices, to understand the residents' preference for the types of sounds in Guilin rural areas and the impact of various sounds on the rural acoustic landscape environment, to provide an important reference for planning and improving the overall environment and acoustic landscape quality of Guilin rural areas.

(2) Method.

The article "Rural Acoustic Landscape Analysis Based on Segmentation and Extraction of Spectral Image Feature Information" was retracted in 2024. Reasons: signs of a paper mill; suspected computer-generated content; unreliable results or conclusions; lack of ethics approval or compliance.

The time of this questionnaire survey is September 15, 2021. The questionnaire survey method is mainly used to investigate rural residents to understand their attention to the overall rural environment in Guilin and their satisfaction with the existing environment, and statistically analyze the main sound types they are most concerned about, analyze their love, and provide a basis for rural sound landscape planning.

(3) Sample characteristics.

In this questionnaire, residents around the project site and future owners of the residential area are the main survey populations, and random sampling methods are used to determine the specific survey objects. A total of 350 questionnaires were sent out during the questionnaire survey, and 328 valid questionnaires were recovered. Through data entry and statistical analysis, the sample characteristics of this survey are shown in Tables 1–4.

### 3.4. Temporal and Spatial Changes of Rural Forest Acoustic Landscape

The most inseparable part of the countryside [29] is the soundscape in the forest, and the most attractive thing is the call of insects and birds. For this reason, this article selects three locations near the countryside in Guilin, Guangxi, namely the foothills, river valleys, and ridges. Statistics of bird calls, insect calls in different seasons, and sound frequencies at different times of the same day, and the data are regularized. The diversity and vertical structure of the three forest plant communities as shown in Table 5.

## 4. An Experimental Analysis of the Soundscape of Guilin Villages in Guangxi Based on the Language Spectrum

### 4.1. Experiment Analysis

(1) Sample analysis.

The following conclusions can be drawn from the sample collection data:

(1) From the analysis of gender, the proportion of men who participated in this questionnaire survey was 46.6%, and the proportion of women was 53.4%. There was little difference in the proportion of men and women.

(2) From the analysis of age distribution, the two age groups of 31–40 and 41–50 have a relatively high proportion of people participating in the survey, and the proportion of people aged 21–30 is also quite large, and those under 20 and over 50. The number of people is small, which can reflect to a certain extent that people in the 21–50 age group pay more attention to the environmental quality of rural construction. But it needs to be stated that there are not many residents over 50 who were invited to participate in this survey, but a considerable number of residents in this age group are not willing to accept the survey.

(3) From the analysis of education level, the proportion of people with a college degree and undergraduate degree and above is relatively high, 33.8% and 24.7%, respectively, and the proportion of high school degree is 19.5%. It can be seen that people with higher education levels pay more attention to the rural environment from another perspective, and it can be seen that people with a high school degree or above are more likely to accept questionnaire surveys and are more willing to provide relevant information and personal opinions.

(4) From the analysis of occupational category, among the surveyed population, office workers accounted for the highest proportion, reaching 48.8%, followed by students and unemployed persons, which were 17.4% and 18.3%, respectively, indicating that office workers are more concerned about the rural areas after getting off work as the main environmental quality issues in relaxing places.

(2) Result analysis.

The article "Rural Acoustic Landscape Analysis Based on Segmentation and Extraction of Spectral Image Feature Information" was retracted in 2024. Reasons: signs of a paper mill; suspected computer-generated content; unreliable results or conclusions; lack of ethics approval or compliance.

By collecting the questionnaire data, we drew statistical graphs from satisfaction and importance based on age, as shown in Figure 6.

From the data in the figure, it can be seen that the villagers' satisfaction and importance with the rural soundscape are extremely high, with 87.19% of satisfaction with the rural soundscape and 92.68% of the emphasis on the rural soundscape. It can be seen that the rural soundscape is a rural construction. To improve the living conditions and living environment of villagers, the construction of a rural soundscape is particularly important.

### 4.2. Field Collection Results of Natural Soundscape in Rural Forests

(1) Seasonal change comparison.

A statistical analysis of the bird community call information in three forests collected in the previous period revealed that there are obvious seasonal changes in frequency and time indicators, as shown in Figure 7.

From the perspective of the length of the bird's song in each plot, the bird's song activity in the three regions showed the same changing trend with the seasonal changes. Reach the maximum value, and reach the minimum value in autumn and winter. It shows that bird song activity is the most abundant in spring, and the weakest in autumn and winter.

Then carry out information extraction and statistics on the insects, and the results are shown in Figure 8.

From the point of view of the frequency of insect sounds in various plots, the center frequency of insects in the piedmont plot is between 5.01 and 6.43 kHz; the center frequency of the insects in the valley plot is between 2.91 and 7.90 kHz; the center frequency of the pest in the ridge plot is between 2.91 and 7.90 kHz and 4.69 and 6.07 kHz. The frequency bandwidth of insect sounds in different seasons also changed. The piedmont and ridge samples had the same changing trend, namely summer > autumn and winter > spring; the frequency bandwidth of the valley samples was spring > summer > autumn and winter. The difference in insect frequency between different seasons indicates that each site has its own unique insect species. The vocal insects adapt to the environment and evolve into different vocal frequency ranges to meet the needs of courtship, and realize intraspecies communication.

(2) Comparison of single-day changes.

The article "Rural Acoustic Landscape Analysis Based on Segmentation and Extraction of Spectral Image Feature Information" was retracted in 2024. Reasons: signs of a paper mill; suspected computer-generated content; unreliable results or conclusions; lack of ethics approval or compliance.

Taking spring as an example, the daily changes in bird song information in a single day are shown in Figure 9.

The duration of the call is an important indicator reflecting the community's call activity. From the point of view of the time of the bird's song, the daily variation of the time of bird's song in the three urban forests in spring showed the same trend, which was basically a “U” shape. There are two peaks in 1 day, which appear at around 5:00 in the morning and around 17:00 in the evening. The time period of the bird's singing in all the sites is basically the same, starting from 5:00 to 7:00 in the morning and ending at 17:00 to 19:00 in the evening, and no bird's singing was observed in other time periods. The diurnal change process of the tweet time indicator in each plot is basically the same, the highest peak of the whole day appears between 5:00 and 7:00 in the early morning, and then gradually weakened. The lowest value of the whole day for the piedmont and ridge samples appeared in the morning from 9:00 to 11:00, while the lowest value of the whole day for the piedmont samples appeared between 13:00 and 15:00 in the afternoon. Until 17:00 in the afternoon, it reached another peak throughout the day, and the activity of bird song increased, and then the activity of bird song stopped until it reappeared at 5:00 in the morning of the next day.

Figure 10 shows the daily changes of insects.

From the point of view of the frequency of insects, the changing trends of insects in the three urban forests have certain differences. From the point of view of the change of the center frequency, the change trend of the foothills and the ridge sample plots is basically the same. The frequency change trend of insect sound in the valley plot is different from that of the other two plots, which mainly manifests in the blank period of chirping from 15:00 to 17:00. From the perspective of bandwidth changes, the ridge and piedmont plots have basically the same range of bandwidth changes, and the bandwidth of the valley plots reaches its peak at night. From the above results, it can be seen that the composition of the song insect community in the valley plots is different from the other two plots. And the composition of songworms in the foothills and ridge plots is similar.

The article "Rural Acoustic Landscape Analysis Based on Segmentation and Extraction of Spectral Image Feature Information" was retracted in 2024. Reasons: signs of a paper mill; suspected computer-generated content; unreliable results or conclusions; lack of ethics approval or compliance.

## 5. Conclusions

This article makes a detailed analysis of the rural acoustic landscape in Guilin, Guangxi, through the segmentation and extraction of the spectral image features. First, the characteristics of the acoustic landscape in the relevant area are investigated on the spot, and then the acoustic landscape research experiment is carried out for the rural and forest modules, and the spectral image is obtained. Carry out Gabor wavelet filtering and segmentation, and extract analysis, and carry out statistical analysis on the average length of the call of insects and birds in the forest, the ratio of singing time, and the relative amount of information. Finally, a questionnaire on the satisfaction and importance of the soundscape of the rural villagers is carried out. Experiments show that the satisfaction of villagers with the soundscape is as high as 87.12%, and the degree of importance is even as high as 92.68%. Therefore, the rural acoustic landscape is a very important part of rural construction. In the future, it will show unique charm.

## Figures and Tables

**Figure 1:** Application areas of soundscape.

**Figure 2:** Schematic diagram of the realization of the spectrogram.

**Figure 3:** Basic representation of the graph: (a) simple undirected graph and (b) matrix representation of undirected graph.

**Figure 4:** Famous scenic spots in Guilin, Guangxi.

**Figure 5:** Landscape of Guilin.

**Figure 6:** Survey results of satisfaction and importance. (a) Survey of villagers' satisfaction. (b) Survey of villagers' attention.

**Figure 7:** Birdsong activity changes in three different seasons. (a) Birdsong duration ratio in different seasons. (B) Birdsong time ratio in different seasons. (c) Ratio of relative information volume of bird song in different seasons.

**Figure 8:** Changes in insect song activity in three different seasons. (a) The time ratio of insects in different seasons. (b) Relative information volume of insects in different seasons.

**Figure 9:** Daily changes of birdsong (a). Daily variation of bird song center frequency (b) day variation, bird's song frequency bandwidth.

**Figure 10:** Daily changes of insects: (a) diurnal variation of the center frequency of insects and (b) daily variation of insects' frequency.

**Table 1:** Sex ratio.

Gender	Rural residents	Residents around the village	Proportion (%)
Male	55	98	46.6
Female	71	104	53.4

The article "Rural Acoustic Landscape Analysis Based on Segmentation and Extraction of Spectral Image Feature Information" was retracted in 2024. Reasons: signs of a paper mill; suspected computer-generated content; unreliable results or conclusions; lack of ethics approval or compliance.

**Table 2:** Proportion of age.

Age	Rural residents	Residents around the village	Proportion (%)
Under 20	12	8	6.1
21–30	23	34	17.4
31–40	45	76	36.9
41–50	38	62	30.5
51–60	5	13	5.5
Over 60 years old	3	9	3.7

**Table 3:** Proportion of educational background.

Education	Rural residents	Residents around the village	Proportion (%)
Elementary school and above	11	18	8.8
Junior high school	16	27	13.1
High school	21	43	19.5
Junior college	46	65	33.8
Bachelor degree and above	32	49	24.7

**Table 4:** Proportion of occupations.

Profession	Rural residents	Residents around the village	Proportion (%)
Student	21	36	17.4
Office worker	63	97	48.8
Unemployed	22	38	18.3
Retiree	9	17	7.9
Other	11	14	7.6

**Table 5:** Species diversity and vertical structure of plant communities in three forests.

Site	Community name	Index of species diversity						Vertical structure of forest		
		Tree layer			Shrub layer					
		H'	E	D	H'	E	D	Number of layers	Gc	Gv
Foothills	Acacia ma Zhan community	1.80	1.64	0.31	1.39	1.66	0.41	4	0.27	40.97
River valley	Green-yellow Pueraria lobata community	2.54	1.20	0.11	1.05	1.85	0.52	4	0.44	48.05
Ridge	Schima superba-Duckfoot community	2.01	1.38	0.18	0.41	4.37	0.84	3	0.20	32.96

## Data Availability

This article does not cover data research. No data were used to support this study.
